This article has been retracted.

# Breast Cancer Exosome-Derived miR-425-5p Induces Cancer-Associated Fibroblast-Like Properties in Human Mammary Fibroblasts by TGF*β*1/ROS Signaling Pathway

**DOI:** 10.1155/2022/5266627

**Published:** 2022-11-30

**Authors:** Yue Zhu, He Dou, Yuqi Liu, Pingyang Yu, Fucheng Li, Youyu Wang, Min Xiao

**Affiliations:** Department of Breast Surgery, Harbin Medical University Cancer Hospital, Harbin, 150081 Heilongjiang, China

## Abstract

The connection between the cellular microenvironment and tumor cells is crucial for tumor progression. However, the process by which normal fibroblasts (NFs) become cancer-associated fibroblasts (CAFs) is unknown, and mounting evidence suggests that some microRNAs (miRNAs) have an important role in converting NFs into CAFs. Breast cancer (BC) has been proven to have enhanced miR-425-5p expression in order to support progression. We discovered that human mammary fibroblasts (HMFs) could uptake BC cell line-derived exosomes to change their properties, promoting the switch to the CAF phenotype and increasing cell motility, as evidenced by an increase in CAF activation-related marker protein expression and cell proliferation, invasion, and migration. Transfection of exosomes is obtained from BC cells, and miR-425-5p inhibitors suppressed the aforementioned effects as well as lowered chemokine levels and gene expression related with proliferation and metastasis. By suppressing the expression of its target gene TGF*β*RII (TGF*β*1 receptor), miR-425-5p enhanced the transition of HMFs to the CAF phenotype. MDA-MB-231 cells and CAFs stimulated by HMF absorption of MDA-MB-23-derived exosomes showed similar proliferation, invasion, migration, and expression of -SMA, FAP, CXCL1, IL-6, TGF*β*1, P21, P27, Ki67, vimentin, E-cadherin, N-cadherin, *α*-catenin, fibronectin, and MMP-2. TGF*β*1 overexpression enhanced ROS production. Finally, we found that HMFs transiently transfected with miR-425-5p can promote tumor growth in vivo. Finally, these findings provide fresh insight on miR-425-5p as an important mediator of the interaction between BC cells and stroma.

## 1. Introduction

Worldwide, breast cancer (BC) is the most often diagnosed malignancy among females. Incidence of breast cancer is rising annually in China, reflecting a recent trend [1]. In recent years, BC mortality has decreased as a result of continuous advancements in early detection, surgical technology, radiotherapy, and chemotherapy, as well as the individualization of endocrine therapy and molecular targeted therapy [2]. However, BC remains the largest cause of cancer-related deaths among women globally. Therefore, it is essential to investigate the pathophysiology of BC.

As a result of a sequentially complex process involving tumor cells, the host, and the tumor microenvironment, tumor recurrence and metastasis have long been important obstacles in cancer therapy and a major focus of cancer research [3]. The tumor microenvironment is a distinguishing feature of the tumor; it is a local homeostatic environment formed of tumor-infiltrated immune cells, stromal cells, and t active mediators released by these cells, all of which play an important role in tumor progression [4]. All fibroblasts found inside and around tumor tissues are referred to as cancer-associated fibroblasts (CAFs), and they are the primary components of the tumor microenvironment, promoting tumor invasion and metastasis via direct or indirect interaction with tumor cells [5]. CAFs can generate a pretransfer microenvironment in a prospective metastatic organ prior to tumor metastasis. It encourages the establishment of metastatic lesions by providing a favorable growing environment for tumor cells that reach specific organs. CAFs play a role in the occurrence and progression of BC. However, their activation and molecular mechanism of action are unknown [6].

Exosomes are membranous nanoscale vesicles found in the extracellular matrix that have a diameter of approximately 30-100 nm. Exosomes' functions in the tumor microenvironment have drawn more attention lately [7]. By transporting miRNAs, long noncoding RNAs (lncRNAs), and messenger RNAs, exosomes can facilitate information exchange between tumor cells and the tumor microenvironment. It suggests that exosomes have potential utility in tumor diagnosis and treatment [8, 9]. miRNAs are a family of noncoding single-stranded RNA molecules between 19 and 22 nucleotides in length that are encoded by endogenous genes. It has been demonstrated that exosomes enhance the transport and transmission of microRNAs between cells and protect them from RNase degradation. When exosomes containing specific miRNAs are picked up by receptor cells, they are able to not only influence gene expression but also directly interact with specific proteins, thereby compromising their biological function [10]. Further research is needed to determine if miRNA transported by tumor cell-derived exosomes enters the tumor microenvironment to regulate CAF activation, thereby driving BC's recurrence and metastasis.

## 2. Materials and Methods

### 2.1. Human Breast Cancer Cell Lines

These human breast cancer cell lines, MDA-MB-231 and BT-549, were obtained from the Shanghai Cell Bank of the Chinese Academy of Sciences for the purpose of this inquiry. They were grown in Dulbecco's Modified Eagle's Medium (DMEM; Hangzhou Sijiqing Bioengineering Materials Co., Ltd., Hangzhou, Zhejiang, China) at a temperature of 37 degrees Celsius and a carbon dioxide concentration of 5%. The medium also contained 10% fetal bovine serum (FBS), 100 units of penicillin per milliliter, and streptomycin (100 micrograms per milliliter). When the confluence reached between 70 and 80 percent, it was necessary to initiate subculture.

### 2.2. Human Mammary Fibroblasts (HMFs)

HMFs that were cultured in DMEM supplemented with 10% FBS, penicillin 100 U/ml, and streptomycin 100 U/ml were provided by ATCC (USA).

### 2.3. Exosome Extraction from Cancer Cells and Serum of BC Patients

After 10 minutes at 3000 rpm, the breast cancer cell culture supernatant was called conditioned medium. MDA-MB-231 and BT-549 exosomes were precipitated using this solution (System Biosciences, Mountain View, CA, USA). ExoQuick-TC exosome pellet was introduced overnight to breast cancer conditioned medium and centrifuged for 30 minutes at 1500 rpm and 5 minutes at 3000 rpm. Exosome pellets were resuspended in 250-500 microliters of cell culture medium and cultured for 72 hours with recipient cells. Exosome-removed medium was recovered after 90 minutes at 25,000 rpm. Serum samples from 67 women with breast cancer and 67 healthy donors were kept at -80°C at the Harbin Medical University Cancer Hospital. There were no significant differences in general characteristics between two groups. The study protocol was approved by the ethics committee of the Harbin Medical University Cancer Hospital. All patients signed the informed consent forms. For 30 minutes at 4°C, the supernatant was centrifuged at 2000 rpm with BC cancer patients' sera and healthy donors' sera. Next, the exosomes were isolated by utilizing the whole exosome isolation reagent (Invitrogen, Carlsbad, CA, USA). An exosome suspension was added to the copper EM grids, and subsequently, the phosphotungstic acid was added. After drying, TEM was utilized to evaluate the shape and size of the exosomes. NanoSight NS300 Nanoparticle Tracking Analyzer (NS300) was used to assess the concentration of exosomes, their size distribution, and their zeta potential (Malvern, UK). Exosome markers TSG101 and HSP70 were used in western blot analysis.

### 2.4. Exosome Uptake Assay

Before beginning the test in 6-well Transwell plates with 0.4 *μ*m pore size filters, an initial step was taken to culture 200,000 MDA-MB-231 and BT49 cells in complete DMEM for 24 hours. This was done before the test ever began (Corning, Sigma-Aldrich). After that, the cells were subjected to some tests. BODIPY TR ceramide was mixed with exosomes from MDA-MB-231 and BT49 cells, which resulted in the incorporation of a dye into the exosomes (Invitrogen). For a full five minutes, the liquid was vigorously stirred in all directions before being drained. The excess dye from the labeled exosomes was removed using an ultracentrifuge that ran at 100,000*g* for an hour at a temperature of 4°C. The exosome pellet was cleaned with PBS three times after it was removed from the ultracentrifuge and placed back into the centrifuge. The pellet was brought back to life with the assistance of PBS. Six hours after the experiment was initiated in PBS and 4% paraformaldehyde, HMF cells were labeled with exosomes that were tagged with BODIPY TR ceramide. Following that, the cells were washed in PBS for a second time (PFA).

### 2.5. Immunofluorescence Staining

For 15 minutes, a 10% formalin (Sigma 47036) solution was added to a 0.5% saponin (Sigma 4771) solution. This fixed the cell cultures. The cells were then washed three times with PBS that did not have any calcium or magnesium in it. The cells were then made more permeable with a 1% Triton X-100 solution, and then, they were washed three times with PBS. The cells were then stained with a blocking buffer made of 1% bovine serum albumin (Sigma) and 1% goat IgG (research on immunology at Jackson). Fluorescence microscopy was done with 50 ng/ml of DAPI from Life Science Technology and monoclonal rabbit or mouse anti-human primary antibodies (-SMA and FAP) (respectively). Between 100 and 110, glycerol was used to seal the slides, and a fluorescence microscope was used to look at them (Olympus).

### 2.6. Fluorescence In Situ Hybridization (FISH)

The 6-FAM-tagged miR-425-5p FISH probe was donated by the Gema Company. Paraformaldehyde was used to fix HMFs, and PBS was used to rinse them. Afterward, the cells were washed with PBS and digested with proteinase K (Sangon, Shanghai) for 5 minutes at 37°C. First, cells were fixed in 1% paraformaldehyde and then denatured with 70%, 85%, and 100% alcohol as specified in the table to dehydrate them. After denatured hybridization solution probes were placed on cell slides and denatured for 3 minutes, the probes were hybridized overnight at 42°C light at 73°C for denatured hybridization solution probes. At 37°C, the slides were pretreated with 0.1 percent NP-40/2SSC and 50 percent formamide/2SSC before being washed at room temperature with DAPI staining solution. This study made use of laser confocal microscopy (LCM) images (Leica, Mannheim, Germany).

### 2.7. Intracellular ROS Levels

The DCFH-DA approach was used in order to get an idea of how the ROS levels have changed relatively. Following transfection, the cells were subjected to a treatment with 10 mmol/L OD DCFH-DA for a period of 30 minutes. Following three washes, the cells were positioned on a fluorescence analyzer (BioTek, USA), and the excitation/emission wavelength was adjusted to 488/525 nm. After then, an assessment of the results was made. The values are shown as a percentage of the relative fluorescence that the control group possessed in comparison to the fluorescence of the experimental group.

### 2.8. Western Blot

In order to separate proteins from exosomes, the Exosomal RNA and Protein Extraction Kit (101Bio) was utilized in a manner that was compliant with the guidelines provided by the manufacturer. The total protein was extracted using RIPA lysis buffer (Beyotime, Shanghai, China), and the protein concentration was determined using a Pierce BCA protein detection kit. This experiment was carried out in Shanghai, China (Thermo Fisher Scientific, Waltham, MA, USA). After loading 25 g of proteins onto a 10% SDS-PAGE gel and separating them using that gel, the proteins were concentrated on a 5% SDS-PAGE gel and then transferred to a polyvinylidene fluoride membrane (Merck Millipore, Billerica, MA, USA). After blocking with 5% bovine serum albumin for 2 hours, anti-TGF1, anti-SMA, anti-FAP, anti-CXCL1, anti-IL-6, anti-TGFRB1II, anti-P21, anti-P27, anti-Ki67, anti-vimentin, and anti-E-cadherin antibodies were injected. Anti-TGF1, anti-SMA, and anti-FAP secondary antibodies were found to be present in the sample after a blocking treatment of 5% bovine serum albumin for two hours. Anti-N-cadherin, anti-catenin, anti-fibronectin, anti-MMP-2, anti-GAPDH, anti-TSG101, and anti-HSP70 antibodies were utilized in this work. All of the antibodies were diluted as directed by the manufacturer, and then, they were incubated at 4 degrees Celsius for one whole night. After that, the primary antibodies were treated with goat anti-rabbit or goat anti-mouse IRDyeTM 800CW secondary antibodies at room temperature for one hour. The Odyssey imaging system was utilized to perform the functions of scanning and processing on the images (LI-COR, Lincoln, NE, USA).

### 2.9. Real-Time PCR (RT-PCR) Analysis

TaqMan miRNA detection technique was utilized in order to provide an accurate reading on the concentrations of miR-425-5p and U6 (Life Technologies, Shanghai, China). Following the completion of reverse transcription, complementary DNA was synthesized with the help of the RT-Master Mix (manufactured by TaKaRa Bio in Shiga, Japan), and RT-PCR with StepOnePlus RT-PCR equipment was used to determine the levels of mRNA expression (Applied Biosystems, Foster City, CA, USA). The primers that were utilized in this research are outlined in Table 1.

### 2.10. Dual-Luciferase Reporter Assay

miR-425-5p was discovered to have the potential to be targets for TargetScan (http://www.targetscan.org/). After transfection, a period of 24 hours was spent using the Dual Luciferase Reporter Assay 22 System to check for the presence of luciferase activity (Promega, Madison, WI, USA).

### 2.11. miR-425, TGF*β*1, and TGF*β*RII Transfection *In Vitro*

From Biomics Biotechnology Co., Ltd., we purchased the miR-425-5p inhibitors and negative control (miR-NC inhibitors), as well as the miR-425-5p mimics and negative control (miR-NC mimics), as well as the TGF1 siRNA (TGF1 knockdown (TGF1-KD)), TGFRII siRNA (TGFRII-KD), and negative control (NC-KD) (Nantong, Jiangsu, China). Both the pcDNA 3.1 vector expressing TGF1 (also known as TGF1 overexpression (TGF1-OE)) and the pcDNA 3.1 vector that did not express TGF1 (NC-OE) were provided by UNIBIO Biotechnology Co., Ltd. (Chongqing, China). They were converted into HMFs by utilizing Lipofectamine 2000 as the transfection agent (Invitrogen, Carlsbad, CA, USA).

### 2.12. Wound Healing Assay

At a temperature of 37 degrees Celsius, cells were grown in 6-well plates in a solution that included 1% fetal bovine serum. The plates were kept at a constant temperature (five times the normal cell population). Once the cells had reached 100% confluence, we were able to successfully streak the monolayer using a pipette tip. After being washed twice in PBS, the cells were grown in culture for forty-eight hours at a temperature of 37 degrees Celsius and 5% carbon dioxide. Under a microscope, pictures were obtained of cells that had been collected at 0 hours and 48 hours after the injury, respectively (TS100-F, Nikon, Tokyo, Japan).

### 2.13. Transwell Invasion Assay

Research on invasion was carried out inside of a chamber that had been coated in Matrigel (BD BioCoat, Corning). While the lower chamber of the Transwell device contained medium containing 10% FBS, the upper chamber was seeded with 1 × 10^4^ cells that were suspended in medium that did not include any serum. In the trials involving invasion, the cells were grown on Matrigel Transwell inserts that had previously been coated in Matrigel. Following an incubation period of 24 hours, the cells that had remained on the upper side of the membrane were eliminated. On the other hand, the cells that had migrated to the bottom surface of the membrane were fixed and stained with 0.1% crystal violet to determine where they were located. Images of the labeled cells were obtained using the microscope (Nikon).

### 2.14. Colony Formation Assay

Before being planted directly into 6-well plates at a density of 5 × 10^2^ cells per well, the cells were digested, and the growth conditions were set at 37 degrees Celsius with 5% carbon dioxide. The cells were grown in culture at a temperature of 37 degrees Celsius with 5% carbon dioxide. After being incubated for two weeks, it was washed with phosphate buffered saline (PBS) three times before being examined (PBS). After being fixed in 100% ethanol for 30 minutes, the cells were then stained with hematoxylin for 20 minutes so that their structure could be seen. This process took place so that the structure of the cells could be seen. In order to obtain an impression of the highest possible quality, the slab was first blasted dry and then dried with a hair drier. A colony is regarded to be a real colony whenever it has more than 50 cells in it.

### 2.15. Animal Experiment

The Institutional Animal Care and Use Committee of Heilongjiang Province, China, gave its approval to every animal study being conducted there. The mice were kept in a sterile environment and fed a special diet that was pathogen-free (SPF) for a period of three to four weeks (Better Biotechnology Co., Ltd., Nanjing, China). The mice's weight ranged from 14 to 28 grams at the beginning of the study (Better Biotechnology Co., Ltd., Nanjing, China). Following the completion of the therapy, the cells were trypsinized and then dissolved in a buffer solution. Each group received an equal amount of cells, which were all adjusted to the same concentration per milliliter of growing medium. The quantity of cells was also kept exactly the same. Cell suspensions were surgically inserted into the thighs of hairless mice (0.5 ml). After that, each of the nudized rats was given food to determine whether or not any tumors had developed. Every week, we measured the volume of the tumor with a caliper to get an accurate reading. In the study of mice that were sacrificed five weeks following the start of the experiment, tumor development curves and tumor weights were produced and compared.

### 2.16. Immunohistochemistry

Following a roasting period of thirty minutes at a temperature of 65 degrees Celsius, tissue slices were removed from the oven, deparaffinized using xylene and alcohol, and then sliced to a thickness of four meters. After the xylene deparaffinization process was complete, the slices were treated with hydrogen peroxide at a concentration of 3 percent in order to suppress the activity of endogenous peroxidase. After antigen retrieval, the sections were treated with bovine serum albumin (BSA) at a concentration of 1 percent in order to reduce nonspecific binding. Using IgG and IgG2a in conjunction with the appropriate secondary antibodies, we were able to detect TGF-1 (1 : 800), B-SMA (1 : 500), vimentin (1 : 400), Ki67 (1600), and CXCL1 (1 : 800). To detect TGF-1 (1 : 800), B-SMA (1 : 500), and vimentin (1 : 400), as well as Ki67 (1600), we used the appropriate secondary antibodies (1600) (1 : 3000). After being stained with DAB and hematoxylin for a considerable amount of time, the slices were evaluated and assessed by two separate observers. The existence of tumor cells as well as the degree of staining was taken into consideration when determining the final grades.

### 2.17. Construction and Verification of Risk Prediction Model

R (v3.6.1) features LASSO regression and multivariate Cox regression analysis. “glmnet” avoided model overfitting with LASSO regression. “Survival's” multivariate analysis determined the model's final variables using LASSO regression. Each patient's risk score was calculated using regression coefficients and gene expression levels. BC patients have prognostic risk scores. We categorized BC patients using the median risk score. Long-term survival rates were compared using Kaplan-Meier curves and the log-rank test. This study used ROC and AUC to evaluate risk models. Gene transcription heatmaps and risk score maps were used to evaluate the model.

### 2.18. Statistical Analysis

During the course of this inquiry, each experiment was carried out using at least three biological replicates. The mean and standard deviation are both shown in the table that is located above. GraphPad Prism8 and SPSS 22.0 were the software packages that were applied in order to carry out statistical analysis (IBM, Armonk, NY, USA). When comparing two groups, the *t*-test for independent samples was utilized; however when comparing several groups, the one-way analysis of variance was utilized. In order to determine whether or not there were any changes that were statistically significant, the Kaplan-Meier curves and the log-rank test were applied to the overall survival analysis. The Pearson correlation test was applied to the data gathered for the investigation of correlation (Pearson correlation coefficient). The two-sided *P* value of 0.05 indicated that there was a difference that may be considered statistically significant (*n* = 3).

## 3. Results

### 3.1. Exosomes Derived from MDA-MB-231 and BT549 Cells Promoted the Transition of HMFs to the CAF Phenotype

Exosomes from MDA-MB-231 and BT549 cells were examined and characterized, indicating that they exhibit a typical membrane structure and diameter of less than 100 nm under TEM (Figures 1(a) and 1(b)). The exosome marker protein TSG101 was significantly increased, and HSP70 was remarkably decreased by western blot (Figure 1(c)). Following that, exosomes from MDA-MB-231 and BT549 cells were cultured with HMFs in an attempt to induce HMFs to acquire the CAF phenotype (Figure 1(d)). The findings demonstrated that HMFs could uptake exosomes from MDA-MB-231 and BT549 cells (Figure 1(e)), and that these HMFs had high levels of *α*-SMA and FAP*α* expression (Figure 1(f)). Therefore, these cells were given the names CAFs(M) and CAFs(B).

### 3.2. miR-425-5p Was Highly Expressed in Exosomes Derived from MDA-MB-231 and BT549 Cells

FISH assay revealed that miR-425-5p (red) was expressed in HMFs, MDA-MB-231, and BT549 cells (Figure 2(a)), but its expression level and number were significantly higher in MDA-MB-231 and BT549 cells than in HMFs (Figure 2(b)). Meanwhile, miR-425-5p expression was noticeably higher in exosomes isolated from MDA-MB-231 and BT549 cells when compared to HMFs (Figure 2(c)). Subsequently, miR-425-5p inhibitors were transfected into MDA-MB-231 and BT549 cells to reduce miR-425-5p expression (Figure 2(d)). After that, to inhibit miR-425-5p expression in CAFs, exosomes were extracted from MDA-MB-231 and BT549 cells that had been transfected with miR-425-5p inhibitors (Figure 2(e)).

### 3.3. miR-425-5p Inhibitors Inhibited the Proliferation, Invasion, and Migration of HMFs Induced by Exosomes

To determine whether exosomes can induce HMFs the switch to CAFS phenotype, we examined the motility of HMFs that had ingested exosomes using the clone formation, Transwell, and cell scratch tests. The results indicated that MDA-MB-231 and BT549 cell exosome-containing HMFs significantly increased proliferation (Figure 3(a)), invasion (Figure 3(c)), and migration (Figure 3(e)). However, HMFs that incorporated exosomes from miR-425-5p inhibitor-transfected MDA-MB-231 and BT549 cells had significantly lower proliferation (Figure 3(b)), invasion (Figure 3(d)), and migration (Figure 3(f)) capacities than HMFs that did not.

### 3.4. Exosomes Derived from BC Cells Accelerated the Transition of HMFs to the CAF Phenotype

We used exosomes derived from miR-425-5p inhibitors transfected MDA-MB-231 and BT549 cells to coincubate with HMFs and detect related gene expression in order to further elucidate the role of miR-425-5p on exosomes secreted by BC cells in the conversion of HMFs to CAF phenotype. The changes in the expression of these genes were compared to those in HMFs treated with nontransfected BC cell exosomes. Western blot and RT-PCR analysis revealed that exosomes from MDA-MB-231 and BT549 cells significantly increased the expression of *α*-SMA and FAP*α* and promoted the levels of CXCL1, TGFB1, and IL-6 in HMFs (Figures 4(a) and 4(b)). However, exosomes from miR-425-5p inhibitor-transfected BC cells decreased the expression of the above genes in HMFs and reversed the effects of exosomes from BC cells on P21, P27, and Ki67 (Figure 4(c)). Four genes, including vimentin, N-cadherin, fibronectin, and MMP2, are expressed more frequently by exosomes from BC cells than two other genes, including *α*-catenin and E-cadherin, in HMFs. These effects were abolished when exosomes from BC cells were transfected with miR-425-5p inhibitors (Figure 4(d)).

### 3.5. Exosomal miR-425-5p Stimulated HMF Switch to the CAF Phenotype

Following that, we would transfect miR-425-5p inhibitors into CAFs that were HMFs ingesting exosomes from MDA-MB-231 cells in order to determine whether exosomal miR-425-5p is the primary factor promoting the HMFs to adopt the CAFS phenotype. The proliferation, invasion, and migration abilities of MDA-MB-231 cells and CAFs were consistent, implying that HMFs ingested exosomes from MDA-MB-231 cells that exhibited distinct CAF phenotype characteristics (Figures 5(a)–5(c)). However, miR-425-5p inhibitors could significantly restrain the proliferation, invasion, and migration of CAFs. The expressions of *α*-SMA, FAP*α*, CXCL1, IL-6, TGF*β*1, P21, P27, Ki67, vimentin, N-cadherin, *α*-catenin, fibronectin, MMP2, and E-cadherin were not significantly different between the CAFs miR-NC and the MDA-MB-231 groups (Figures 5(d)–5(g)). On the contrary, transfection of CAFs with miR-425-5p inhibitors results in a decrease in *α*-SMA, FAP*α*, CXCL1, IL-6, TGF*β*1, Ki67, vimentin, N-cadherin, fibronectin, and MMP2 and an increase in P21, P27, E-cadherin, and *α*-catenin (Figures 5(d)–5(g)).

### 3.6. Exosomal miR-425-5p Stimulated Tumor Growth *In Vivo*

Tumor formation experiments in naked mice revealed that MDA-MB-231 cells transfected with miR-425-5p mimics were significantly more tumorigenic than MDA-MB-231 cells or MDA-MB-231 cells transfected with miR-425-5p inhibitors. However, there was no difference between MDA-MB-231 cells transfected with miR-NC and MDA-MB-231 cells transfected with miR-425-5p inhibitors in terms of their capacity to cause tumors (Figures 6(a)–6(c)). After that, HMFs fed exosomes derived from MDA-MB-231 cells demonstrated oncogenicity *in vitro* (Figure 6(d)). Transfection of CAFs with miR-425-5p mimics increased the oncogenicity *in vitro*, whereas transfection with miR-425-5p inhibitors decreased the oncogenicity *in vitro* (Figures 6(e) and 6(f)). IHC staining revealed that miR-425-5p inhibitors suppressed the intensity of TGF*β*1, *α*-SMA, vimentin, Ki67, and CXCL1 expressions in tumor tissues of mice injected with MDA-MB-231 cells (Figure 6(g)). Similarly, miR-425-5p mimics further strengthened the expression intensity of TGF*β*1, *α*-SMA, vimentin, Ki67, and CXCL1 in tumor tissues of mice injected with CAFs derived from MDA-MB-231 cells, while miR-425-5p inhibitors suppressed the expression intensity of TGF*β*1, *α*-SMA, vimentin, Ki67, and CXCL1 to the greatest extent possible in tumor tissues (Figure 6(h)).

### 3.7. miR-425-5p Upregulated TGF*β*1 Expression via Inhibiting TGF*β*RII to Promote HMFs Switch to the CAF Phenotype and Increasing ROS Level

According to the TargetScan database, miR-425-5p was targeting TGF*β*RII, also known as the TGF*β*1 receptor (Figure 7(a)). miR-425-5p mimics increased miR-425-5p expression while decreasing TGF*β*RII expression when transfected into HMFs, whereas miR-425-5p inhibitors decreased miR-425-5p expression while increasing TGFRII expression (Figures 7(b) and 7(c)). The dual-luciferase reporter assay revealed that cells cotransfected with TGF*β*RII-wt and miR-425-5p mimics had significantly decreased luciferase activity, while cells cotransfected with TGFRII-mut and miR-425-5p mimics remained substantially unchanged (Figure 7(d)). Next, miR-425-5p mimics transfection increased TGF*β*1 expression while transfection of its inhibitors suppressed TGF*β*1 expression (Figures 7(e) and 7(f)). In order to detect changes in the expression of genes related to CAF phenotype transition, chemotaxis, and inflammation, siRNA-TGF*β*RII was transfected into HMFs to inhibit its expression (Figure 7(g)). Our findings showed that miR-425-5p mimics, or siRNA-TGF*β*RII treated HMFs, BC cells, and exosomes secreted by these cells were highly expressed in *α*-SMA and FAP*α* (Figure 7(h)). In addition, miR-425-5p mimics treatment HMFs and siRNA-TGF*β*RII transfection in HMFs could elevate the expression of CXCL1, IL-6, and TGF*β*1 similar to what occurs in exosomes from BC cells (Figure 7(i)). Then, we found that exosomes from BC cells, miR-425-5p mimics, and TGF*β*RII knockout all have the same ability to promote proliferation and invasion of HMFs (Figure 7(j)). After inhibiting TGF*β*1 expression in HMFs (Figures 8(a) and 8(b)), the expression of *α*-SMA, FAP*α*, CXCL1, IL-6, and TGF*β*1 was significantly decreased (Figures 8(c) and 8(d)). On the other hand, TGF*β*1 promoted the expression of *α*-SMA, FAP*α*, CXCL1, and IL-6 (Figures 8(c) and 8(d)). We obtained 141 intersected target genes from two database (TargetScan and starBase) (Figure 8(e) and Sup Table 1 and Table 2). Based on the STRING website (https://cn.string-db.org/), STRING analysis showed that a protein-protein interaction (PPI) network included TGF*β*1, TGF*β*RII, and ROS (Figure 8(f)). Our results showed that TGF*β*1 increased ROS levels (Figure 8(g)).

### 3.8. Construction of Prognostic Model for Exosomal miR-425-5p in BC Patients

We discovered that functional miR-425-5p was substantially expressed in exosomes from BC cells. As a result, we studied the differential expression of miR-425-5p in human serum exosomes. Serum samples from 67 cancer patients and healthy donors were used to isolate and identify exosomes. The shape of exosomes from BC patients is illustrated in Figure 9(a). The exosomes' size range was within 200 nm, with a median of 112 nm (Figure 9(b)). Exosome marker protein TSG101 significantly increased, while exosome marker protein HSP70 significantly decreased, according to a western blot analysis (Figure 9(c)). miR-425-5p was substantially expressed in exosomes from serum of BC patients as compared to healthy donors, as shown by RT-PCR (Figure 9(d)). “miR-425-5p high” patients with BC were those whose exosomal miR-425-5p expression levels were at or above the exosomal miR-425-5p median value (3.5). We observed a favorable correlation between exosomal miR-425-5p expression and tumor size, TNM staging, and histological grade, but not with age (Table 2). BC patients with exosomal miR-425-5p^high^ had a poor prognosis (Figure 9(e)). The LASSO regression analysis was performed, and the above four variables, including age, tumor size, TNM staging, and histological grade, were selected for the multivariate Cox regression analysis (Figures 9(f) and 9(g)). According to the findings, the ROC curve's AUC for these four parameters was 0.835 (Figure 9(h)). Based on the median value of exosomal miR-425-5p, the risk score of each patient was calculated, and the patients were divided into high- and low-risk groups, suggesting that the highly expressed miR-425-5p group has a higher risk score (Figure 9(i)). Kaplan-Meier curve demonstrated that the prediction model was more effective, and BC patients in the high-risk category had a lower OS rate (Figure 9(j)). Independent prognostic analysis revealed a significant correlation between the 4-factor risk signature and the OS of BC patients by the univariate Cox regression (*P* < 0.001, HR = 1.370, 95% CI = 1.182-1.586) and the multivariate Cox regression analyses (*P* < 0.001, HR = 1.346, 95% CI = 1.190-1.523) (Figures 9(k) and 9(l)). A nomogram was built that integrated clinicopathological features with risk score, risk-group, and exosomal_miR-425-5p expression to predict the survival features of BC patients, as shown in Figure 9(m).

## 4. Discussion

Tumor cells and stromal cells both contribute to the formation of the tumor microenvironment by the secretion of extracellular matrix components such as fibronectin, collagen, proteoglycans, glycoproteins, growth factors, and matrix metalloproteinases [7, 11]. The interaction of epithelial and mesenchymal cells is required for the conversion of NFs to CAFs [12]. CAFs as extracellular matrix are one of the most abundant nonlymphocyte components of tumor microenvironment. CAFs can regulate tumor cell metabolism, migration, stem cell phenotype, and extracellular matrix restructuring, which in turn promotes tumor angiogenesis, proliferation, invasion, and metastasis of tumor cells [5]. To determine whether breast cancer-derived exosomes may successfully promote the conversion of HMFs to CAFs, it is crucial to examine whether the HMFs that take up exosomes generated by breast cancer cells exhibit the phenotypic and motor features of CAFs. Our findings indicate that HMFs consuming tumor-secreted exosomes have enhanced cell proliferation, motility, and invasion capacities as well as high levels of *α*-SMA and FAP*α*, which are classical biomarkers for CAFs. High expression of *α*-SMA and FAP*α* is closely associated with poor prognosis in tumor patients. This suggests that exosomes secreted by breast cancer cells can promote the transformation of fibroblasts into CAFs.

In recent years, studies have found that miRNAs loaded with breast cancer cell-derived exosomes may influence the tumor microenvironment and consequently affect the invasion and metastasis of breast cancer [13]. It was reported that exosomal miR-21 promoted cisplatin resistance in esophageal squamous cell carcinoma [14]. For example, miRNA dysregulation in melanoma has been shown to promote CAF activation via induction of epithelial-mesenchymal transition (EMT), which in turn alters the secretory phenotype of CAFs in the stroma [15]. miR-425-5p may act on oncogene in breast cancer given that it has been demonstrated to promote tumor progression and that it is significantly upregulated in breast cancer [16], gastric cancer [17], lung cancer [18], and other tumors. In addition, an interesting study confirmed that the highly expressed miR-425-5p in pancreatic cancer was significantly positively correlated with the expression of inflammatory factor (IL-23) [19]. In summary, these studies point to miR-425-5p as a comprehensive factor that can regulate the pathophysiology of cancer. In this study, we found that miR-425-5p was not only expressed in breast cancer cells but also expressed in HMFs. What distinguishes HMFs from breast cancer cells is that miR-425-5p expression is significantly lower, suggesting that miR-425-5p may be a “bridge” molecule between HMFs and CAFs. After that, miR-425-5p inhibitors were transfected into breast cancer cells; the exosomes of the above cells were then retaken by HMFs, demonstrating a significant increase in cell proliferation, invasion, and migration. However, we found that miR-425-5p inhibitor uptake significantly reduced the increased proliferation, migration, and invasion induced by exosomes derived from breast cancer cells. This reversely demonstrated that miR-425-5p could be transmitted to HMFs through exosomes to increase cell motility. In light of the diverse phenotypic characteristics of CAFs, the epithelial-mesenchymal transition-associated proteins vimentin, E-cadherin, and N-cadherin; migration invasion-related proteins *α*-catenin, fibronectin, and MMP2 [20]; chemokine CXCL1, inflammatory factor IL-6, and TGF*β*1 [21]; and proliferation-associated proteins P21, P27, and Ki67 were selected as judge indicators for the conversion of HMFs to CAFs [22]. The results indicated that uptake of exosomes derived from breast cancer cells increased expression of CXCL1, IL-6, TGF*β*1, Ki67, vimentin, N-cadherin, fibronectin, and MMP2 in HMFs and inhibited the expression of P21, P27, *α*-catenin, and E-cadherin expressions. Based on the above experimental results, we determined that breast cancer cell sourced-exosomes can promote the phenotype transformation of HMFs to CAFs. However, miR-425-5p inhibitors greatly decreased the ability of breast cancer cell-derived exosomes to induce the transformation of HMFs into CAF phenotypes. We transfected miR-425-5p inhibitors into HMFs uptaking BC cell-derived exosomes and found that the cell motility and phenotypic characteristics were consistent with those of HMFs uptaking BC cell-derived exosomes transfected with miR-425-5p inhibitors. These provide additional evidence that BC cell-derived exosomes can promote the conversion of HMFs to CAFs by delivering miR-425-5p.

It is a classic mechanism for miRNA to act on the occurrence and development of tumors by inhibiting its downstream target genes [23]. Here, we found that TGF*β*RII is a target gene of miR-425-5p and can be significantly inhibited by it. TGF*β*RII is one of the receptors for TGF*β*1, and it is the only one that can independently accept TGF*β*1 in the absence of another ligand, thus affecting the activation of TGF*β* signaling pathway, which is involved in cell growth, apoptosis, differentiation, proliferation, migration, and epithelial-mesenchymal transformation, among other functions [24]. It reported that TGF*β*1 induced oxidative stress to generate ROS production and that TGF*β*1 was the most effective cytokine for inducing the transformation of NFs to CAFs [25, 26]. It is reported that TGF*β*1 induces ROS production to promote EMT development and cancer progression [27–29]. Interestingly, many studies have been reported on the role of TGF*β*RII in inhibiting and promoting cancer [30, 31]. This study focuses for the first time on the relationship between exosome-derived miRNAs and the TGF*β*1/ROS pathway during the phenotypic transformation of CAFs. In this study, we found that TGF*β*RII knockout can promote the phenotypic transformation of HMFs to CAFs, which is analogous to the function of TGF*β*1 expression in this process. Our understanding of this is as follows: TGF*β*1 binds TGF*β*RII in large quantities, which leads to decreased expression of TGF*β*RII in cells, but activates TGF*β* signal to increase TGF*β*1 release; TGF*β*1 overexpression generated ROS, thus promoting the transformation of HMFs to CAF phenotype. Our results also showed that miR-425-5p mimics upregulated TGF*β*1 expression and promoted the phenotype transformation from HMFs to CAFs.

Finally, we established a prognostic risk model by identifying miR-425-5p expression in plasma exosomes of BC patients and found that patients with high miR-425-5p expression in exosomes had a significantly better prognostic. In addition, miR-425-5p is associated with poor prognosis in BC patients. It showed that exosome-derived miR-425-5p offers fresh insights into the occurrence and development of BC and provides a potential novel target for molecular therapy for patients with BC.

However, in this study, the mechanism and action of exosome-derived miR-425-3p in BC is only described at the molecular level, and the transcriptional level (e.g., transcriptome sequencing) of patient blood samples was not explored. We will keep increasing the sample size in subsequent studies and look into its function in immune activity in the tumor microenvironment.

In conclusion, the involvement of miR-425-5p in reprogramming the microenvironment via inhibition of TGF*β*RII expression and production of ROS to activate TGF*β*1/ROS signaling pathway, thereby promoting tumor growth in normal fibroblasts via EMT, migration, and invasion, in addition to its tumor-growth role (Figure 10), endows this miRNA with a significant therapeutic potential in breast cancer.

## Figures and Tables

**Figure 1:** Exosomes derived from MDA-MB-231 and BT549 cells promoted the transition of HMFs to the CAF phenotype. (a) Exosome identification by TEM. (b) Size distribution of MDA-MB-231- and BT549-derived exosome diameters. (c) Detection of TSG101 and HSP70 protein expression by western blot. (d) Human mammary fibroblasts. (e) Exosome uptake assay observed HMFs taking in MDA-MB-231- and BT549-derived exosomes. (f) Immunofluorescence staining observed the expression of *α*-SMA and FAP*α* in HMFs uptaking MDA-MB-231 and BT549 cell-derived exosomes.

**Figure 2:** miR-425-5p was highly expressed in exosomes derived from MDA-MB-231 and BT549 cells. (a) The location of miR-425-5p in HMFs, MDA-MB-231, and BT549 cells by FISH. (b) The level of miR-425-5p in HMFs, MDA-MB-231, and BT549 cells by RT-PCR. (c) The level of miR-425-5p in HMFs, MDA-MB-231, and BT549 cell-derived exosomes by RT-PCR. (d) miR-425-5p inhibitors were transfected into MDA-MB-231 and BT549 cells to detect the level of miR-425-5p by RT-PCR. (e) The level of miR-425-5p in HMFs uptaking exosomes from miR-425-5p transfected MDA-MB-231 and BT549 cells by RT-PCR. Experimental data presented as means ± standard deviation. Experiment was repeated 3 times. ^∗∗^*P* < 0.01 compared with the HMFs, HMFs_exo, control, and CAFs(M/B) groups.

**Figure 3:** BC cell-derived exosomes induced proliferation, invasion, and migration of HMFs and expedited HMF switch to CAF phenotype. In HMFs uptaking exosomes from miR-425-5p inhibitors transfected MDA-MB-231 and BT549 cells, the cell proliferation (a, b), invasion (c, d), and migration (e, f) were detected by clone formation, Transwell, and scratch-wound assays. Experimental data presented as means ± standard deviation. Experiment was repeated 3 times. ^∗∗^*P* < 0.01 compared with the control group. ^##^*P* < 0.01 compared with the exo_miR-NC inhibitor group.

**Figure 4:** BC cell-derived exosomes induced protein expression to expedite HMF switch to CAF phenotype. In HMFs uptaking exosomes from miR-425-5p inhibitors transfected MDA-MB-231 and BT549 cells, the expression of *α*-SMA and FAP*α* (a), CXCL1, TGF*β*1, and IL6 (b), P21, P27, and Ki67 (c), and vimentin, E-cadherin, N-cadherin, *α*-catenin, fibronectin, and MMP2 (d) were detected by RT-PCR and western blot assays. Experimental data presented as means ± standard deviation. Experiment was repeated 3 times. ^∗∗^*P* < 0.01 compared with the control group. ^##^*P* < 0.01 compared with the exo_miR-NC inhibitor group.

**Figure 5:** Exosomal miR-425-5p stimulated HMF switch to CAF phenotype. In miR-425-5p transfected CAFs (HMFs uptaking exosomes from MDA-MB-231 cells), cell proliferation (a), invasion (b), migration (c), the expression of *α*-SMA and FAP*α* (d), CXCL1, TGF*β*1, and IL6 (e), P21, P27, and Ki67 (f), and vimentin, E-cadherin, N-cadherin, *α*-catenin, fibronectin, and MMP2 (g) were detected by RT-PCR and western blot assays. Experimental data presented as means ± standard deviation. Experiment was repeated 3 times. ^∗∗^*P* < 0.01 compared with the MDA-MB-231 group. ^##^*P* < 0.01 compared with the CAF miR-NC group.

**Figure 6:** Exosomal miR-425-5p stimulated tumor growth *in vivo*. (a) Tumors in mice transplanted with miR-NC transfected MDA-MB-231 cells and miR-425-5p mimics/or inhibitors transfected MDA-MB-231 cells. (b) Growth curve of tumors in different groups. (c) Tumor weight in different groups. (d) Tumors in mice transplanted with miR-NC transfected CAFs and miR-425-5p mimics/or inhibitors transfected CAFs. (e) Growth curve of tumors in different groups. (f) Tumor weight in different groups. (g, h) IHC staining showed the expression of TGF*β*1, *α*-SMA, vimentin, Ki67, and CXCL1 in different groups. Experimental data presented as means ± standard deviation. Experiment was repeated 3 times. ^∗∗^*P* < 0.01 compared with the MDA-MB-231 miR-NC/CAFs miR-NC group. ^##^*P* < 0.01 compared with the MDA-MB-231 mimics/CAF mimics group.

**Figure 7:** miR-425-5p upregulated TGF*β*1 expression via targeting TGF*β*RII-inhibition to promote HMF switch to CAF phenotype. (a) TargetScan database showing a target gene of miR-425-5p was TGF*β*RII. The expression level of miR-425-5p (b) and TGF*β*RII (c) in miR-425-5p mimics/inhibitors transfected HMFs by RT-PCR. (d) Dual-luciferase reporter assay detected the luciferase activity in cells cotransfected with TGF*β*RII-wt/or mut and miR-425-5p mimics. (e, f) TGF*β*1 expression in miR-425-5p mimics/or inhibitors transfected HMFs was detected by RT-PCR and western blot assays. (g) The expression of TGF*β*RII in si-TGF*β*RII transfected HMFs was detected by RT-PCR. The expression of *α*-SMA and FAP*α* (h), CXCL1, IL8, and IL6 (i), and cell proliferation (j) were detected by RT-PCR and western blot, clone formation assays in HMFs uptaking MDA-MB-231-derived exosomes. Experimental data presented as means ± standard deviation. Experiment was repeated 3 times. ^∗∗^*P* < 0.01 compared with the miR-NC mimics, miR-425-5p mimics, NC-KD, and control group. ^##^*P* < 0.01 compared with the miR-NC inhibitors and NC-OE groups.

**Figure 8:** TGF*β*1 promoted ROS production to promote HMF switch to CAF phenotype. siRNA-TGF*β*1 and overexpression-TGF*β*1 were transfected into HMFs; the expression TGF*β*1 (a, b), *α*-SMA and FAP*α* (c), and CXCL1, IL-8, and IL-6 (d) were detected by RT-PCR and western blot assays. (e) Venn analysis of overlapping genes. (f) A PPI network based on STRING website. (g) ROS level. Experimental data presented as means ± standard deviation. Experiment was repeated 3 times. ^∗∗^*P* < 0.01 compared with the NC-KD group. ^##^*P* < 0.01 compared with the NC-OE group.

**Figure 9:** Construction of prognostic model for exosomal miR-425-5p in BC patients. (a) Exosome from blood of BC patient identification by TEM. (b) Size distribution of MDA-MB-231- and BT549-derived exosome diameters. (c) Detection of TSG101 and HSP70 protein expression by western blot. (d) The mRNA level of miR-425-5p was detected in exosomes from blood between healthy donors and BC patients. (e) Kaplan-Meier survival analysis for miR-425-5p expression in exosomes from blood of BC patients. (f, g) LASSO Cox analysis identified 4 factors correlated with the overall survival. (h) The ROC curve showed that the AUC of the 4-factors prognostic model was 0.835. (i) Risk score distribution, survival overview, and the heatmap showing the expression profiles of miR-425-5p from exosomes in the high- and low-risk groups. (j) The patients in the high-risk group exhibited a worse overall survival than those in the low-risk group. (k) Independent prognostic analysis showed that the 4-factor risk signature was significantly correlated with the OS of BC patients by a univariate Cox regression analysis. (l) Independent prognostic analysis showed that the 4-factor risk signature was significantly correlated with the OS of BC patients by a multivariate Cox regression analysis. (m) The nomogram of risk score and clinical characteristics. LASSO: least absolute shrinkage and selection operator; ROC: receiver operating characteristic; AUC: area under curve; OS: overall survival. Experimental data presented as means ± standard deviation. Experiment was repeated 3 times. ^∗∗^*P* < 0.01 compared with the normal group.

**Figure 10:** The schematic diagram depicts the regulatory mechanism of exosomes deliver miR-425-5p in HMF switch to CAF phenotype. Exosomal miR-425-5p promoted HMF switch to CAF phenotype via inhibiting TGF*β*RII expression to activate TGF*β*1 signaling pathway, thereby playing tumor-promoting abilities in normal fibroblasts.

**Table 1:** The sequences of the primers.

Gene	Forward (5′-3′)	Reverse (5′-3′)
miR-425-5p	AGGATAGTCCATGTTAGGAA	AGCCCTGCAAAGACTGGTAGCG
TGF*β*1	ATGCTGTAGTAGTAGGTGTT	CTGTGTCTCAATACGTCT
TGF*β*RII	TGTGTCACTGTACCTGTAA	ACTGTGTGTAAGTGTAAA
Vimentin	GCAACTGTGTCCACAA	CGAGCTGTGTTGTATGCATGT
E-cadherin	GTGTAACTGAATGCTAGCTAA	CCCATGTACCATGTAACA
N-cadherin	TTGCAGCTGCAATCGTAGTG	ACTCTGTGATCTGACTGAA
*α*-Catenin	CCGCTAGTGTAAGCCAAATGCC	CGTGACAATGTACCTGAAAC
Fibronectin	GCAACGCATGTCTGTGTAACA	AATGACATGGTAGAACAA
MMP2	CCATGACGATATGTAGTAG	ACGTGACATGTCTGCTGAA
CXCL1	TTAACCTCCGTGTAAATGCG	ATGTGACGTGCATGACTG
IL-6	GTAATGTGACGCGTGTAAAAAC	CCGACGTGGCTCCATAAACAA
P27	AACGTGTAGTGTAGGATA	CGTAGCTACCTAGATCCGTG
Ki67	TAACGCGCTTGTGTAGTGA	GTAGGTAAGGTTCCAGTA
P21	AACAAATGGACGTGCAAA	TAAGAGCTGGCTGTGTCCT
U6	TTCGGTTAAATTGCCCCAGAC	CGCACCTAAGGCGAGTA
GAPDH	CCCGCAGTTAGCCAACTTCTCG	CGTCTTACACACAGGTAACGAA

**Table 2:** Clinicopathological variables and exosomal miR-425-5p expression in 67 breast cancer patients.

Variables	Cases (*n* = 67)	Exosomal miR-425-5p		*χ* ^2^	*P* value
		Low	High		
Ages (years)				1.697	0.193
≤ 50	28	16	12		
> 50	39	16	23		
Tumor size (cm)				27.771	0.000^∗^
≤ 2	28	24	4		
>2	39	8	31		
TNM staging				5.280	0.022^∗^
I-II	30	19	11		
III-IV	37	13	24		
Histological grade				17.541	0.000^∗^
Well differentiated	9	8	1		
Moderately differentiated	24	16	8		
Poorly differentiated	34	8	26		

## Data Availability

The data will be available upon reasonable requests from the corresponding author.
